# Image Analysis of TVCDS in Infertile Patients with Polycystic Ovary Syndrome

**DOI:** 10.1155/2022/1234983

**Published:** 2022-06-17

**Authors:** Hongju Duan, Shihua Luo, Yang Yu, Qiaohua Yan

**Affiliations:** Yunnan Medical Health College, Kunming 650033, Yunnan, China

## Abstract

In order to analyze and examine the TVCDS images of infertile patients, this paper conducted an in-depth study based on the symptoms of polycystic ovary syndrome. Through the sample size estimation method, mathematical analysis, and other methods, the image examination of the polycystic ovary in TVCDS was successfully analyzed. 86 cases of infertile patients with PCS were divided into a control group treated with clomiphene alone and an observation group treated with clomiphene combined with TCM periodic therapy, with 43 patients in each group. The therapeutic effects of the two groups were compared and analyzed. Results show that the treatment effective rate and pregnancy success rate of the observation group were 95.35% and 88.37%, respectively, and those of the control group were 83.72% and 76.74%, respectively. The difference between the two groups was statistically significant (*P* < 0.05). It was understood that the main pathogenesis of polycystic ovary syndrome is the abnormal balance of kidney, *qi*, and blood meridians. Thus, the balance of kidney-anemone-chong Ren-uprisal is broken and the result is infertility symptoms or irregular menstruation. After a study on TVCDS in infertile patients, it was observed that the levels of progesterone (P) and luteinizing hormone (LH) in patients with irregular menstruation were significantly increased. The increase was higher than that in the control group, with an overall negative rate of 4.00%, compared with 18.00% of the control group, showing a significant difference. It also indicates that TVCDS image examination has a very significant effect on improving menstrual irregularities and reducing the incidence of adverse reactions.

## 1. Introduction

Polycystic ovary syndrome is the main cause of infertility in women, including endocrine problem symptoms with abnormal glucose metabolism and reproductive dysfunction, with an incidence of about 6%. Polycystic ovary syndrome is a common clinical gynecological disease but is also an important cause of infertility in patients, often leading to a poor ovulation cycle and abnormal hormone levels. Western medicine treatment is mainly hormone-based, where the purpose is to regulate the hormone level, promote normal ovulation, and so on. Traditional Chinese medicine believes that polycystic ovary syndrome can be included in the amenorrhea infertility category. It is a multicausal and multisymptomatic disease mainly caused by follicular developmental disorders. It is manifested as oligomenorrhea or amenorrhea, hyperandrogenemia, infertility, obesity, recurrent miscarriage, gestational diabetes mellitus, hypertension, increased incidence of metabolic syndrome, and cardiovascular and cerebrovascular diseases. Due to abnormal ovarian function and hormone levels in the body, it is not easy for a woman having this type to conceive and she is more prone to miscarriage after pregnancy. At the same time, the risk of developing gestational diabetes, gestational hypertension, and other obstetric complications increased compared with other women. Women with PCOS may appear to have a lot of follicles, but they just do not ovulate. It is like seeing a bunch of “grapes” hanging from the vine, which is tempting, but the bunch of “grapes” has never been ripe. If you give it a little fertilizer to help them grow up faster (ovulation induction), it is very likely that this bunch of “grapes” will ripen dozens of times, causing ovarian hyperstimulation syndrome (OHSS). This disease should not be underestimated. Once it occurs, it can range from abdominal distention, abdominal pain, nausea, and vomiting to pleural effusion, ascites, and thromboembolism and can even be life-threatening in more serious cases. OHSS does not occur naturally; it can only happen during ovulation induction. Therefore, one of the effects of PCOS on IVF treatment is an increased risk of OHSS. However, professional reproductive doctors in regular hospitals will take various measures to control ovulation and minimize the chance of OHSS. TVCDS examination of infertile patients with polycystic ovary syndrome showed that ovarian volume, interstitial area, number of follicles, and total ovarian blood flow velocity signal intensity increased significantly and vascular resistance decreased. The pathogenesis of infertility with polycystic ovary syndrome is complex, and the clinical manifestations are rich and varied. TVCDS is widely used in gynecology examination means, with high-resolution probe frequency characteristics. The probe can be close to the cervix and vaginal dome, convenient for close observation of the ovary and uterus and for a clear display of reproductive organ lesions. Factors leading to ovulation disorders are shown in Figure 1. The imaging of the observation group showed a bilateral ovarian volume increase, and the maximum follicle diameter was 0.74 cm. There were more than 10 small follicles in the cortex ranging from 2 to 7.4 mm in diameter. In addition, the endometrial thickness was lower, and OV, SA, FN, and TA were higher than that in the control group (*P* < 0.05). In conclusion, ovarian volume, ovarian interstitial area number, and ovarian total area increased significantly. However, the bilateral ovarian volume of the control group was normal without the above changes, which can provide a valuable reference for the identification and diagnosis of infertility with polycystic ovary syndrome. At the same time, the ovarian and uterine artery blood flow of women of normal childbearing age was regulated by sex hormone levels and showed typical periodic changes.

## 2. Literature Review

Naseri R. et al. said that the polycystic ovary syndrome (PCOS) is the most common gynecological endocrine disease, affecting 8% to 30% of women of childbearing age [1]. Basak R. et al. believed that the main clinical manifestations of PCOS were amenorrhea, infertility, hirsute acne, etc., biochemical characteristics were increased levels of androgen, luteinizing hormone (LH), etc., and B-ultrasound showed polycystic changes and enlargement of bilateral ovaries. In addition to reproductive dysfunction, patients with insulin resistance, abnormal glucose metabolism, and dyslipidemia are at an increased risk of developing type 2 diabetes and cardiovascular diseases [2]. Ni Z. et al. believed that it seriously harms women's health, and the main clinical manifestations and biochemical characteristics are highly heterogeneous, which makes TCM have some difficulties in clinical syndrome differentiation, and it also affects the accuracy of syndrome differentiation and the pertinence of dispatching prescription drugs to a certain extent. It is the core of the TCM theory. Syndrome element is the smallest unit of syndrome, which constitutes the minimum unit of the syndrome [3]. Fehintola A. et al. indicated that syndrome elements can be divided into disease-location syndrome elements (such as liver, spleen, and kidney) and disease-type syndrome elements (such as blood stasis, qi deficiency, and qi stagnation). The syndrome differentiation method based on syndrome elements is easy to master clinically and can improve the accuracy, standardization, and repeatability of syndrome differentiation, thus improving the level of clinical diagnosis and treatment [4]. Therefore, Taman et al. believed that patients with congenital genital malformation, adrenal disease, thyroid disease, pituitary tumor, hyperprolactinemia, and other related symptoms caused by endocrine diseases had primary organic lesions in the heart, lung, liver, kidney, and other important organs [5]. Dorgham N. et al. believed that infertile patients with polycystic ovary syndrome had endocrine and metabolic disorders, with high levels of luteinizing hormone. Under the regulation of estrogen, ovarian blood vessels dilated significantly, so vascular resistance decreased and the blood flow speed increased [6]. Therefore, Li N. et al., in addition to accumulated teaching experience, focused on observing the changes of ovarian hemodynamics and signal intensity in the TVCDS examination of suspected infertility patients with polycystic ovary syndrome, which was conducive to the definite diagnosis of the disease [7]. Jena Saubhag A. et al. said that world epidemiological studies have shown that the incidence of female infertility has increased, causing problems for the patients' family harmony. Polycystic ovary infertility accounts for the majority of infertility causes [8]. Adebisi O. et al. believed that at the present stage, patients in the treatment group were 26–34 years old, with an average age of (25.2 ± 3.2) years; menstruation lasted from 1 to 7 months, with a mean of (2.54 ± 1.25) months; control patients were 24–35 years old, with a mean age of (64.2 ± 3.2) years; menstrual cycles ranged from 1 to 6 months, with an average menstrual cycle of (4.25 ± 1.25) months [9]. Almeshari W. et al. believed that the main symptoms and signs of the laboratory examination results of B-ultrasonography in the symptoms related to sparse ovulation or anovulation; the late menstruation is up to 501 cases, accounting for 96.72%; 171 cases (33.1%) suffered from infertility, 157 were amenorrhea cases (30.31%), and there were 52 cases (10.04) of irregular vaginal bleeding [10].

## 3. Research Method

### 3.1. Sample Size Estimation Method

In this paper, 84 symptoms and signs related to PSCO constant witness were selected as possible variables. In implicit variable analysis, the sample size should be 5–10 times of the variable, so the sample size should be estimated in at least 420 cases. Cycle therapy of the traditional Chinese medicine is an artificial cycle therapy, which is mainly the use of the traditional Chinese medicine theory combined with the modern medical menstrual cycle of ovarian function changes in the law, in the treatment of menstrual cycle according to the fluctuation of Yin and Yang qi and blood changes with drugs. In this study, patients in the treatment group received TCM periodic therapy, and patients in the control group received clomiphene treatment [11]. Genetic factors are considered to be one of the major pathogenesis of PCOS. Studies have found that the pathogenesis of PCOS has familial aggregation and is mainly inherited in an autosomal dominant manner, which is more likely to occur in first-degree relatives. The massive release of gonadotropin-releasing hormone (GnRH) leads to an increase in luteinizing hormone (LH). The release of LH can increase androgen levels. High levels of LH inhibit the function of follicle-stimulating hormone (FSH), arresting follicle development, and combine with high androgen levels, eventually leading to polycystic ovarian changes. Abnormal and immature oocytes are exposed to high levels of androgens in the follicular fluid, blocking the development of dominant follicles, causing follicle growth arrest or even atresia, and the endometrium has no progesterone resistance due to continuous stimulation of estrogen levels, increasing the risk of endometrial cancer.  Figure 2 shows the number of patients with recent polycystic disease and the number of cured patients, and the change curve of partial PCOS is shown in Figure 3. After treatment, the total effective rate of the treatment group was higher than that of the control group, and the serum follicle-stimulating hormone (FSH), luteinizing hormone (LH), and testosterone level (T) of the treatment group was lower than those of the control group; the difference was statistically significant. It is fully confirmed that TCM periodic therapy can help patients' endocrine, promote their return to the normal level, and improve the patient's ovulation rate and pregnancy rate. All patients signed informed consent, and patients with reproductive system malformation and immune infertility were excluded [12]. Based on the random number table method, 86 patients were randomly divided into the control group treated with clomiphene alone and the observation group treated with clomiphene combined with TCM periodic therapy, with 43 patients in each group. There was no significant difference in age distribution, infertility time, and other basic data between the two groups (*P* > 0.05).

### 3.2. Survey Study

On the basis of previous studies, a PCOS information collection form was developed, including filling in instructions, diagnosis of informed consent, inclusion and exclusion criteria, basic information, brief medical history, physical examination, TCM symptoms and signs, TCM syndrome differentiation, syndrome elements examination, and laboratory results [13]. The information of the four diagnoses was collected by uniformly trained physicians, and the extracted symptoms and signs were differentiated according to syndrome differentiation according to the clinical experience of 2 gynecologists above the deputy director of traditional Chinese medicine, as the syndrome elements of PCOS. Under normal circumstances, a woman's ovaries produce a group of eggs every month, but most of them are eliminated, and eventually, only one mature egg is released into the fallopian tube during ovulation. Due to genetic, environmental, and other factors, some women are more likely to produce “androgens” (i.e., high male hormones) in their bodies. The accumulation of excess androgens in the ovaries will make the eggs unable to mature or release, so they have to stay in the ovaries and cannot get out. “Polycystic”, repeatedly, the “power” of androgens will become larger and larger, which will lead to many major health problems. Polycystic ovary syndrome is a complex endocrine and metabolic disease common in women of reproductive age due to chronic ovulation and excess androgen production in women. As a feature, the main symptoms are irregular produce cycle, infertility, hirsutism, or acne, which is the most common project disorder in women. Polycystic ovary syndrome occurs in women between the ages of 20–40 years and its clinical presentation varies. Excess androgen is the basic feature of polycystic ovary syndrome, including testosterone, free testosterone, diluted diketone and corpus luteum, production hormone, luteinizing hormone, follicle-stimulating hormone ratio, free estradiol, estrone, fasting insulin, and other hormones, whose levels are obviously increased. Each completed information collection form has been audited by the subject leader. Fasting venous blood was taken from the second to fourth day of the menstrual cycle to detect six sexual hormones. The irregular blood could be detected at any time and the OGTT test was performed. Gynecological B-ultrasonography was performed on the third to fifth day of the menstrual cycle for those with regular menstruation, and abdominal ultrasonography was performed for those without sex. Other patients opted for transvaginal ultrasound, which recorded the ovarian volume and the number of sinus follicles in each ovary [14].  Figure 4 shows the curve of the human body size and number of follicles. It is hard to diagnose just based on symptoms. TVCDS is widely used in gynecology examination means, with high resolution probe frequency characteristics. The probe can be close to the cervix and vaginal dome, convenient for close observation of the ovary and uterus and for a clear display of reproductive organ lesions.  Figure 5 shows TVCDS examination method study in the observation group, and imaging shows the bilateral ovarian volume increase, with the maximum follicle diameter of 0.74 cm [15].

### 3.3. Mathematical Statistics

The frequency of renal deficiency in the infertile group was significantly higher than that in the infertile group (*P* < 0.05), and the frequency of fire or heat was significantly lower than that in the infertile group (*P* < 0.05). There was no significant difference in the frequency of other syndromes between the two groups (*P* > 0.05)(*P* > 0.05) [16]. Academicians believe that women suffer from polycystic ovary syndrome due to “genes” but so far there is no clear cause. The mainstream community believes that polycystic ovary syndrome may be a metabolic disease, which was previously thought to be caused by the abnormal secretion of male hormones or gonadotropins in the ovaries. In recent years, studies have also found that it is also related to excessive insulin caused by anti-islet and excessive insulin leads to more and more insulin secretion in the body, which stimulates ovarian cells, produces more male hormones, and affects the ovary. Persistent endometrial hyperplasia can easily lead to endometrial cancer. Women who have no plan for pregnancy can take oral contraceptives or use progesterone regularly to peel off the endometrial regularly. Patients with polycystic ovary syndrome and obesity are also more likely to suffer from hyperlipidemia, hypertension, and cardiovascular disease than the general population. For these patients, it is very important to adjust living habits and lose weight; regular blood tests before meals are also necessary to check blood cholesterol, triglycerides, and blood sugar levels . SPSS14.0 analysis was used to prove the data in this day, and the counting data were expressed as percentage of example (%) and the method was used to test. The measurement data are expressed by item inspection. *P* < 0.05 was considered as a statistically significant difference [17] (see Figure 6). The size and shape of the uterus and ovary were observed, and the endometrial thickness was measured at the position 1 cm away from the fundus, that is, the distance between the echo of the myometrium at the junction between the endometrium and the front wall of the uterine cavity. Then, color Doppler blood flow imaging was carried out, and the included angle of blood flow sound velocity was calibrated to below 60. Attention was given to rotate and adjust the direction of the probe to obtain the best image [18].

## 4. Results and Analysis

The distribution of syndrome elements in the group with and without high androgen clinical manifestations and the frequency of phlegm and dampness in the group with high androgen clinical manifestations were higher than those in the non-androgen group of clinical trials (*P* < 0.05) [19]. The frequency of blood stasis was significantly lower than that of the group without clinical manifestations of high androgen (*P* < 0.05). The treatment effect and pregnancy success rate of the two groups were compared and analyzed. Among them, the evaluation basis of therapeutic effects is as follows: after treatment, menstrual volume at the end of menstruation was significantly reduced and ovulation dysfunction disappeared, indicating a significant effect; the clinical symptoms of the patients improved significantly after treatment, indicating effectiveness; after treatment, the symptoms of patients were not improved and even the trend of aggravation was indicated as invalid [20]. PCOS is a common complication in women of reproductive age. Its incidence is related to a certain genetic abnormality, and living habits also affect the degree of manifestation of polycystic disease. It can cause symptoms such as high male hormones in the blood of women (clinical symptoms such as hirsutism, acne, and baldness), irregular menstruation, obesity, infertility, or easy miscarriage. For polycystic patients, it is very important to change lifestyle habits to keep the weight within the ideal range (BMI < 24), and it can also reduce the complications of other symptoms (such as hyperlipidemia and diabetes). Infertility caused by polycystic ovaries can be overcome with medicine, but the medical community is still working hard to prevent the occurrence of the polycystic ovary. The main pathogenesis of polycystic ovary syndrome is abnormal balance of kidney, qi and blood, and channels and collaterals. Thus, the balance of kidney - anemone - chong Ren - uprisal is broken and irregular menstruation and infertility symptoms happen. Therefore, the TCM treatment of this disease is mainly based on the tonifying kidney. PSV and EDV are parameters in hemodynamic ultrasound that reflect the blood flow velocity of the ovarian artery. RI and PI are the reflection of the ovarian artery resistance parameters. The results of this study showed that the PSV and EDV blood flow signal intensity in the observation group was higher than that in the control group, and RI and PI were lower than that in the control group (*P* < 0.05), suggesting that ovarian blood flow velocity increased and vascular resistance decreased in infertile patients causing the Stein–Leventhal syndrome. Patients with PCOS infertility have endocrine and metabolic disorders, with high levels of luteinizing hormone. Under the regulation of estrogen, ovarian blood vessels dilate significantly, so vascular resistance decreases and blood flow speed accelerates [21]. The results are shown in Figures 7 and 8. Therefore, when clinical TVCDS examination is performed on suspected infertile patients with polycystic ovary syndrome, the observation of changes in ovarian hemodynamics and signal intensity is emphasized, which is conducive to the definite diagnosis of the disease.

## 5. Conclusion

Women's menstruation is a physiological process. Long-term irregular menstruation or unstable menstrual volume is caused by abnormal function of the hypothalamic-pituitary-ovarian axis, which has a serious impact on women. In this study, estradiol valerate is mainly used in the treatment of female menstruation to simulate the changes in ovarian secretion when menstruation occurs, so as to establish a new menstrual cycle and achieve the purpose of improving women's menstruation. Clinically, more than 70% of polycystic ovary syndrome patients are accompanied by delayed menstruation. The clinical manifestations are oligomenorrhea, amenorrhea, etc. The occurrence of these symptoms may be caused by polycystic ovary syndrome. Patients may have amenorrhea due to ovulatory dysfunction and may even have abnormal menstrual periods due to a drop in hormone levels. These manifestations require timely treatment. Polycystic ovary is called a polycystic ovary if more than 12 small follicles are found in one ovary or both ovaries during B-ultrasound in the follicular phase, that is, follicles between 0.2 and 0.9 cm. If the normal menstruation is normal and there is normal ovulation, it will not affect the pregnancy. The appearance of polycystic ovaries during simple B-ultrasound indicates that the fertility is relatively strong, which is a normal phenomenon and does not require treatment. However, when doing B-ultrasound, it can be found that the ovaries are polycystic, and at the same time, irregular menstruation or no menstruation occurred for a long time, and acne and hirsutism appeared, which is polycystic ovary syndrome. This disease is lifelong. Sexual diseases are also difficult to cure. Congenital insufficiency of kidney gas or acquired injury of kidney gas, deficiency of kidney gas cannot get sperm into pregnancy, and can cause infertility. Lack of kidney Yang, Ming men fire failure, chong Ren lost in warm, cell palace cold can cause cold infertility. The occurrence frequency of fire heat in the infertile group was low, indicating that the infertility caused by fire heat was relatively rare in clinic. The levels of progesterone (P) and luteinizing hormone (LH) in the observation group were significantly higher than those in the control group. The total incidence of adverse reactions was 4.00% compared with 18.00% in the control group, which was significantly different. It indicates that TVCDS image examination has a very significant effect on improving menstrual irregularities and reducing the incidence of adverse reactions. This suggests that ovarian volume, interstitial area, number of follicles, and total ovarian area increase significantly in infertile patients with PCOS. However, the bilateral ovarian volume of the control group was normal without the above changes, which can provide a valuable reference for the identification and diagnosis of infertile patients with polycystic ovary syndrome. At the same time, the ovarian and uterine artery blood flow of women of normal childbearing age was regulated by sex hormone levels and showed typical periodic changes.

## Figures and Tables

**Figure 1:** Factors that lead to ovulation disorders.

**Figure 2:** Number of recent patients with polycystic syndrome and cured patients.

**Figure 3:** Partial PCOS curve.

**Figure 4:** Human body size and a follicle number curve.

**Figure 5:** TVCDS check means.

**Figure 6:** Regional polycystic infertility rate.

**Figure 7:** Vascular resistance diagram of endocrine and ovarian vessels.

**Figure 8:** Patients with polycystic infertility symptoms.

## Data Availability

The data used to support the findings of this study are available from the corresponding author upon request.
